# Analysis of Sentiment and Personalised Recommendation in Musical Performance

**DOI:** 10.1155/2022/2778181

**Published:** 2022-06-02

**Authors:** Dan Wang

**Affiliations:** Huaihua University, School of Music and Dance, Huaihua, Hunan Province 418000, China

## Abstract

Music performance research is a comprehensive study of aspects such as emotional analysis and personalisation in music performance, which help to add richness and creativity to the art of music performance. The labels in this paper in collaborative annotation contain rich personalised descriptive information as well as item content information and can therefore be used to help provide better recommendations. The algorithm is based on bipartite graph node structure similarity and restarted random wandering. It analyses the connection between users, items, and tags in the music social network, firstly constructs the adjacency relationship between music and tags, obtains the music recommendation list and indirectly associated music collection, then fuses the results according to the proposed algorithm, and reorders them to obtain the final recommendation list, thus realising the personalised music recommendation algorithm. The experiments show that the proposed method can meet the personalised demand of users for music on this dataset.

## 1. Introduction

As an important vehicle to showcase the charm of music, music performance art can play a role in enriching the form of musical expression and enhancing the connotation of music performance art [1]. It is also an important vehicle for the expression of music and the enhancement of its connotation. The addition of modern music aesthetics to music performance art can, on the one hand, inject strong expressive power into the art and, on the other hand, bring audiences the ultimate visual and audio enjoyment [2]. The study of modern music aesthetics can contribute to the progress and innovation of music performance art and can also attract more people to the art of music performance, thus contributing to the overall development of the music industry. The study of contemporary music aesthetics is therefore important and needs to be implemented as soon as possible [3].

Music aesthetics has a long history and culture. As early as the ancient Greeks, Pythagoras and Plato noted the therapeutic effect of musical aesthetics on the human mood and how the good or bad character of music could make the listener's soul beautiful or ugly [4]. However, they were constrained by their time to explain the reason for this, thus giving a strong mystical dimension to musical aesthetics [5]. As the times have developed, modern musical aesthetics is no longer unknown and has extended into two directions of study, psychological and social [6]. The psychological dimension of modern music aesthetics follows the same direction as that of the ancient Greeks, in that it relates to the psychological knowledge of people's reactions to listening to music in order to find the differences between the general mental activity and the psychological activity of music aesthetics [7]. The social dimension of modern music aesthetics is to relate music to social issues, for example, by analysing the social issues of the time in which the music was composed through the context in which it was written [8].

The art of music performance is a secondary activity of music creation. For the performer, it is a way of presenting the full range of musical achievements in the form of vocal, instrumental, and dramatic music, thus expressing the ideological content of the music [9]. For the listener, the art of music performance is not only an essential way of appreciating and understanding the content and form of music but also a way of identifying and recognising the different interpretations of music by different music performers through the comparison of different performances. At the same time, different performance styles, genres, and techniques will enhance the audience's understanding of the music, thus giving them a sense of thought and emotional resonance [10].

With the development of information technology and the Internet, people are gradually moving from an era of information scarcity to an era of information overload. In this era, both information consumers and information producers have encountered great challenges: for information consumers, it is very difficult to find the information they are interested in from a large amount of information; according to the different technologies used, music recommendation systems can be broadly divided into three categories: content-based recommendation algorithms, collaborative filtering recommendation algorithms, and hybrid recommendation algorithms [11]. Content-based recommendation algorithms select appropriate items for recommendation based on the item's attribute associations, the location of the item, the item's metainformation (keywords describing the item, in the case of music, album, genre, artist name, lyrics, audio, etc. [12]), and the user's history [13]. However, the keywords used by the user do not correspond well to the item description tags, and converting audio information to digital information leads to increased computation and response time. This content-based approach also ignores the similarity of interests between different users and is therefore not well suited to community-based networks [14].

However, model-based algorithms are usually very time-consuming to build and update, and they do not cover all users as well as memory-based algorithms [15]. Collaborative filtering recommendation algorithms and content-based recommendation algorithms each have their own focus and shortcomings [16]. The main idea of the hybrid recommendation algorithm is to combine the above two recommendation methods in order to make full use of the information of users and resources. One of the most influential systems is the Fab [17] from Stanford University. There are also many research results in China in this area [18].

In order to achieve the recommendation of music that users may be interested in, this paper makes use of the information provided in social networks as much as possible and explores the intrinsic connection between users, tags, and items [19]. First, the two bipartite graphs of the user song and tag song are used to build the adjacency matrices of items and tags, respectively; then, the user vector is used to perform a restart-type random walk on the two adjacency matrices to obtain the list of related songs and related tags of the user; finally, the first *N* tags of the related tag list are selected. Finally, the top *N* tags of the relevant tag list are selected and the indirectly associated music set is mined from the tag-song relationship. The indirectly associated music set is used to adjust the ranking of the user's relevant song list and recommend the items with high scores to the user. Experimentation on the corpus collected by Last.fm shows that the proposed method performs better than the collaborative filtering algorithm [20].

## 2. Theory Related to Recommendation Algorithms

In traditional collaborative recommendation systems, users are required to give explicit ratings to indicate their liking of the item, and these ratings are generally limited and discrete. The memory-based algorithm can be divided into user-based and item-based collaborative filtering recommendation algorithms.

The user-based collaborative filtering algorithm is based on the assumption that if users rate some items similarly, they will also rate other items similarly. The algorithm approximates the target user's ratings of an item based on the ratings of the target user's nearest neighbours (the most similar users). Define the target user *a* and its unrated item *i*. Then, predict *a*'s rating of *I* as follows:

(1) $$\begin{array}{c} p_{a,i}={\bar{r}}_{a}+\frac{\sum_{u=1}^{K}\left(r_{u,i}-{\bar{r}}_{u}\right)\omega_{a,u}}{\sum_{u=1}^{N}\omega_{a,u}}, \end{array}$$

where *r*_*u*,*i*_ denotes the rating of item *i* by the user *u*, ${\bar{r}}_{u}$ and *r*-*u* denote the average rating of the user *a* and the user *u*, respectively, and *ω*_*a*,*u*_ denotes the similarity between the user *u* and the user *a*.

In contrast, the item-based collaborative filtering algorithm considers that there is similarity in users' ratings of different items, and when it is necessary to estimate users' ratings of an item, it can be estimated using users' ratings of several similar items of that item, as shown in the following equation:

(2) $$\begin{array}{c} p_{a,i}={\bar{r}}_{i}+\frac{\sum_{k=1}^{M}\left(r_{a,k}-{\bar{r}}_{k}\right)\omega_{i,k}}{\sum_{k=1}^{M}\omega_{i,k}}, \end{array}$$

where ${\bar{r}}_{k}$ denotes the average score of the item *I* and *ω*_*i*,*k*_ denotes the similarity between the item *i* and the item *k*. In practical commercial applications, the user-based collaborative filtering algorithm is more efficient than the item-based one. In the corpus used in this paper, the number of songs is much larger than the number of users, and for efficiency, the user-based collaborative filtering algorithm is used as the comparison experiment in this paper.

Regardless of the method, the similarity between items and items or between users and users is calculated when predicting the score. There are many ways to calculate the similarity, but the most popular Pearson correlation coefficient is used in this paper, as shown in the following equation:

(3) $$\begin{array}{c} \omega_{a,u}=\frac{\sum_{i=1}^{M}\left(r_{a,i}-{\bar{r}}_{a}\right)\left(r_{u,i}-{\bar{r}}_{u}\right)}{\sqrt{\sum_{i\in I_{a}\cap I_{u}}{\left(r_{a,i}-{\bar{r}}_{a}\right)}^{2}}\sqrt{\sum_{i\in I_{a}\cap I_{u}}{\left(r_{u,i}-{\bar{r}}_{u}\right)}^{2}}}. \end{array}$$

Obviously, in this algorithm, the more items the users rate together, the higher the similarity. However, assuming that both users only rate the same item, the similarity between the two users calculated by this method is very large, which is not reasonable. In order to reduce this situation, it is set that if the number of items jointly rated by two users, *n*, is less than the threshold *Tr*, then the similarity is multiplied by a factor. In addition, this paper uses the *k*-nearest neighbour method to select similar users of the target user.

The dataset used in this paper is based on the number of times a user listens to a song to indicate how much the user likes a particular song, rather than an explicit rating of the item by the user based on their own liking. In order to fuse the label information, the similarity between users *ω*(*UTr*)_*a*,*u*_, *u*, and *αω*(*UTr*)_*a*,*u*_ is first calculated from the number of times a user listens to a song and the user's label, respectively, and the sum of the two is used as *ω*_*a*,*u*_, as shown in the following equation:

(4) $$\begin{array}{c} \omega_{a,u}=\alpha \omega {\left(UTr\right)}_{a,u}+\beta \omega {\left(UTg\right)}_{a,u}, \end{array}$$

where *α* + *β* = 1.

## 3. Music Recommendation Algorithm

We present the personalised music recommendation algorithm based on latent semantic mining in the user-tag item starting with the two-part diagram, followed by the latent semantic mining algorithm on the three-part diagram.

### 3.1. Correlation Matrix for Two-Part Diagrams

The relationship between a user and a song can be represented as a bipartite graph *G*1 = <*U*, *E*1>, where the set of vertices *U* represents the set of users in the recommender system, and if user *u*_*i*_ has listened to music *Tr*_*j*_, then an edge *Tr*_*j*_ is created between *u*_*i*_ and the number of times the user has listened to the music. Similarly, the relationship between a user and a label can be represented as a bipartite graph *G*2 = <*U*, *E*2>, where an edge is created between the user and the label if there is a connection between the two. Then, the above two bipartite graphs are projected onto the dimensions of music and tag, respectively, and the weights of the edges between the node *i* and the node *j* after the projection represent the similarity between music (tag) *i* and music (tag) *j*. In this paper, the cosine method is chosen to calculate the node similarity, as shown in the following equation:

(5) $$\begin{array}{c} \omega_{i,j}=\frac{\left|\Gamma_{i}\cap \Gamma_{j}\right|}{\sqrt{\left|\Gamma_{i}\right|X\left|\Gamma_{j}\right|}}, \end{array}$$

where Γ_*i*_ is the set of neighbouring nodes of the node *i* before projection.

### 3.2. Recommendation Algorithms Based on Bipartite Graphs

The two-part graph-based recommendation algorithm estimates the relationship between users and items by ranking them. The algorithm represents a user node as a vector, and each dimension of the vector represents an item in the association graph, whose value in this paper records the number of times the user has listened to the music node or has used the tag, i.e., the user's interest in the song or tag. The algorithm uses the random walk with the restart model (RWR) to predict the interest of the user node *u*_*i*_ in node *Tr*_*j*_ or *Tg*_*j*_. The random walk starts from the user node and traverses the whole graph. For any node, the traverser walks with probability 1 − *a* to the node's neighbouring nodes and returns to the node with probability *a* to start the walk again. Each walk yields a probability distribution that describes the probability that each vertex in the graph will be visited. This probability distribution is used as input for the next walk, and the process is iterated over and over. The probability distribution of this point converges when the previous and next probability distributions are the same or essentially similar. After convergence, a stable probability distribution is obtained, which represents the closeness of the user node to the project.

For the bipartite graph composed of user music, definition **U**_*i*_^*tr*^ is a user query vector built from the record of songs listened to by user *u*_*i*_ in the training set, with playcount denoting the number of times the user listened to the *j*th song, and vector *q*_*i*_ is a normalized vector of **U**_*i*_^*tr*^. Each dimensional element of **U**_*i*_^*tr*^ is defined as shown in the following equation:

(6) $$\begin{array}{c} U_{i}^{tr}=\left\{\begin{array}{c} \text{playcount,}\\ 0. \end{array}\right) \end{array}$$

The purpose of the algorithm is to obtain the music items that are most closely related to the user. If the association graph consists of *N* music nodes, the steady-state probability vector **S**_*i*_^*tr*^=[*S*_*i*_^*tr*^(1), *S*_*i*_^*tr*^(2),…, *S*_*i*_^*tr*^(*N*)] corresponding to *u*_*i*_ is the desired one. After experimental verification, *S*_*i*_^*tr*^ has reached convergence when the number of iterations *t* = 10.

### 3.3. Semantic Mining

Each user has their own interests, which are presented in the form of tags on their personal description page. When a user listens to music, social media allows the user to tag the item, and these tags reveal the user's perception of the item they are currently listening to. Over time, users' tags become richer and more sophisticated; in addition, a single item can be tagged by multiple users. For these reasons, there is a phenomenon in social media where different users have different perceptions of the same music item and where multiple tags for a music item may imply the same meaning. Therefore, we propose the following idea: a bipartite graph can be used to mine tags with the same meaning; the more tags an item and a user have in common (including similar meanings), the more the user is associated with the item. The workflow of a personalised recommendation system based on potential semantic mining in user-tag music is shown in Figure 1.

The same algorithm is applied to the user-tag bipartite graph to obtain a list of tags associated with the current user. **S**_*i*_^*tg*^=[*S*_*i*_^*tg*^(1), *S*_*i*_^*tg*^(2),…, *S*_*i*_^*tg*^(*M*)]. The difference is that the list of tags obtained by this method does not exclude the tags used by the user itself, as these tags clearly indicate the interests of the user. Then, the *N* tags with the highest relevance to the user are selected and the music collection corresponding to these tags is extracted, which is defined as the “indirectly related music collection.” Finally, the list of song recommendations is modified and reordered according to the song collection, and the final recommendation results are obtained. The weighting equation (7) is used to readjust the song weights:

(7) $$\begin{array}{c} \omega_{i,j}^{\prime }=\omega_{i,j}\times \left(1+\frac{m}{p}\right), \end{array}$$

where *m* denotes the number of occurrences of an identical song corresponding to different tags and *p* denotes the ranking position of the song in the intersection set (an intersection set is an ordered set of intersections between a collection of indirectly associated music and the original recommendation list by weight). It reflects two ideas: (1) the music corresponding to the tag that is more associated with the user is also more associated with the user; (2) multiple tags associated with the user correspond to the same music, which is more associated with the user. After adjusting the weights, the music is reordered in descending order of weights and top *N* is rerecommended to users. After counting the data in the dataset, the average number of tags per user is 10. Therefore, the number of relevant tags for a user should be more than the number of tags owned by the user itself, so as to obtain extended tags and more information. However, the more relevant the tags are, the more computationally intensive the algorithm will be and the efficiency of the algorithm will be reduced. Based on the above two points, 30 tags with high relevance to the user will be selected for the calculation in this paper [21, 22].

## 4. Analysis of Experimental Results

### 4.1. Last.fm Dataset

Last.fm is a musical social network that allows users to create their own personal pages, make friends, add tags, and record the names and times they listen to songs. In 2008, the Computer Science and Technology Laboratory at the University of Glasgow collected and extracted a corpus from the music community site Last.fm and made it publicly available for scholarly research. The corpus contains 3,148 users, 30,520 songs, 12,565 tags, and 5,616 friendships among 3,148 users. This paper is a study of this corpus [23, 24].

For each user, all songs in the corpus are divided into three parts: the training set, which is 80% of the songs that the user has listened to; the test set, which is 20% of the songs that the user has listened to; and the set of songs that the user has not listened to.

### 4.2. Experimental Results and Analysis

In this paper, we compare the user-based collaborative filtering recommendation algorithm with the bipartite graph-based collaborative recommendation algorithm, where each set of experiments is designed to compare the recommendation algorithm with the simple model after adding the label information adjustment. The experiments using the user-music relationship and the experiments adjusted by adding user label information are denoted by *UT*_*r*_ and *UT*_*r*_*Tg*, respectively. The experiments use P@N as the evaluation index, and for each method, P@5, P@10, P@20, P@100, and P@200 are calculated for the comparison experiments.  Table 1 shows a comparison of the effectiveness of different recommendation algorithms using Last.fm as the dataset [25, 26].

As shown in the last row of Table 1, the two-part graph-based collaborative recommendation algorithm is significantly more effective than the user-based collaborative filtering algorithm in the same dataset, and the RWR algorithm with user labels is optimal. This is because the user-based recommendation algorithm only considers the relevance of the users and ignores the relevance between items.

As shown in Figure 2, after the user-based collaborative filtering algorithm is adjusted with the tag information, the overall recommendation effect does not improve, but the recommendation accuracy rate decreases. The reason for this is that although there are 12565 tags in the dataset, the average number of tags per user is 10 according to the experimental statistics. This means that there are very few edges in the user-tag bipartite graph, making the correlation between users obtained from this bipartite graph very small. When a simple weighted sum is applied to the user association matrix obtained from the user-music bipartite graph, the degree of association between users who are already closely related is reduced to some extent, resulting in a decrease in recommendation accuracy. This is a good algorithm if the density of user labels grows with time. In short, social tagging is still a hot topic and a focus of research.

For the improved bipartite graph-based collaborative recommendation algorithm, the accuracy of the recommendations was improved by adding label information and reordering the recommendations, but the effect was not very obvious. The user's browsing habits are mainly focused on the first 20 items in the return list, and the items after that are rarely noticed by the user, so the main goal of this algorithm is to improve the accuracy of the first 20 items in the recommendation list. As can be seen from Figure 3, the algorithm in this paper mainly improves P@10. This is due to the nature of the dataset used. Last.fm has a large number of users and songs, but users rarely tag themselves and their songs, so there are even fewer suitable tags that can accurately locate users and songs. The density of user tags and music tags in the dataset is 4.6 × 10^−4^ and 3.2 × 10^−4^, respectively, making the social tagging information sparse and inevitably mixed with some noisy tags. This makes the application of socially annotated information more difficult. Despite this, the proposed algorithm improves the recommendation results, and as time goes by and the user information and social labeling information become richer, personalised recommendations using community network graphs will be more in line with the interests of users.

As shown in Figure 4, in terms of computational efficiency, given the association matrix TR, the recommendation algorithm based on social annotation and bipartite graphs can obtain a recommendation in *O*(*n*^2^) time with a small number of iterations. However, one of the problems with this algorithm is that if one node in the association matrix TR is updated, the whole association matrix needs to be updated, which will consume *O*(*n*^2^) time.

## 5. Conclusions

The aesthetics of modern music is mainly presented through the art of music performance, which, on the one hand, allows the listener to gain knowledge of the music by learning about its creator and the context in which it was created. On the other hand, music as an emotional carrier carries the full emotion of the music creator, and by listening to music, listeners can have a spiritual resonance with the music creator across generations. In this paper, the bipartite graph-based collaborative recommendation algorithm is further improved by mining the underlying semantics to make more accurate music recommendations. The results of the comparison with the user-based collaborative filtering algorithm and the bipartite graph-based collaborative recommendation algorithm on the same dataset show that this method is a good strategy for personalised recommendation, especially with the development of Web 2.0 and the increase of tags, this method will show a greater advantage.

## Figures and Tables

**Figure 1:** Flowchart of the user-tag-music-based recommendation algorithm.

**Figure 2:** Effect of different music recommendations.

**Figure 3:** Distribution of different levels of music appreciation.

**Figure 4:** Correlation matrix of different music recommendations.

**Table 1:** Comparison of the experimental results of the RWR and CF algorithms.

Method	Specific methods	MAP	P@5	P@10	P@20	P@100	P@200
CF	*UT*_*r*_	0.031	0.142	0.124	0.091	0.047	0.035
	*UT*_*r*_ *Tg*	0.021	0.1101	0.0801	0.0701	0.0385	0.0247

RWR	*UT*_*r*_	0.1024	0.2415	0.3102	0.4412	0.3254	0.2091
	*UT*_*r*_ *Tg*	0.1021	0.2102	0.3251	0.4127	0.3524	0.2021

## Data Availability

The experimental data used to support the findings of this study are available from the corresponding author upon request.
